# Observation of Curative Effect of Trimetazidine Combined with Metoprolol in Elderly Patients with Coronary Heart Disease Complicated with Heart Failure and the Effect of Myocardial Remodeling by Integrated Traditional Chinese and Western Medicine

This article has been retracted.

**DOI:** 10.1155/2022/6098799

**Published:** 2022-09-30

**Authors:** Yingyi Lu, Fenglian Wang, Haoxuan Ni, Ying Sun, Hailing Shi

**Affiliations:** ^1^Shanghai University of Traditional Chinese Medicine Affiliated Hospital of Traditional Chinese Medicine, Shanghai University of Traditional Chinese Medicine, Shanghai, 200336 Shanghai, China; ^2^Shijiazhuang Great Wall Hospital of Integrated Traditional Chinese and Western Medicine-Hebei Province Second Hospital Medical Union, Shijiazhuang, 050035 Hebei, China; ^3^Naval Characteristic Medical Center, Shanghai, 200433 Shanghai, China; ^4^Naval Characteristic Medical Center, Shanghai, 200052 Shanghai, China

## Abstract

Diabetic retinopathy (DR) is the most common complication of diabetes and is often characterized by damage to retinal vascular microcirculation, resulting in retinal exudation, hemorrhage, fibrosis, and neovascularization. With the aging of my country's population, the incidence of DR is increasing year by year, and it has become one of the main blinding eye diseases in ophthalmic diseases also tends to be younger. So far, although the pathogenesis of DR is not completely clear, scholars generally believe that DR is based on the disorder of glucose metabolism, causing changes in the microcirculation of ocular tissues, nerves, and blood vessels, resulting in chronic damage to the nutrition and visual function of the eye disease. In order to explore the demand for cardiovascular disease treatment, make up for the lack of chronic diseases affecting people's physical harm, and improve the success rate of cardiovascular disease treatment, a method to observe the efficacy and myocardial remodeling of trimetazidine combined with metoprolol in elderly patients with coronary heart disease and heart failure based on integrated traditional Chinese and Western medicine was proposed. 54 elderly people over 60 years old are afraid of cardiovascular disease and take active protection. A method based on observation of integrated traditional Chinese and Western medicine was proposed, and at the same time, an intelligent medical monitoring system was constructed to better study, observe, and improve the efficacy of trimetazidine combined with metoprolol in elderly patients with coronary heart disease, heart failure, and myocardial impact of refactoring. The results of the study show that trimetazidine has a good clinical effect on ischemic cardiomyopathy heart failure based on the observation of integrated traditional Chinese and Western medicine.

## 1. Introduction

Cardiovascular and other chronic diseases are relatively common, and they are also a special disease with very high mortality and high medical costs. The occurrence of these diseases is mainly a comprehensive symptom of myocardial systolic or diastolic dysfunction caused by various reasons. In other words, it can also be said to be a progressive syndrome caused by human ventricular dysfunction and pathological remodeling [1]. Diabetic retinopathy can cause severe vision impairment and even blindness. Early studies classified and graded diabetic retinopathy based on the severity of retinal vasculopathy because the contents of the intraretinal vasculature were easily visualized. Based on the level of microvascular degeneration and associated ischemic damage, diabetic retinopathy is broadly classified into two stages: nonproliferative diabetic retinopathy (NPDR) and proliferative diabetic retinopathy (PDR). In the NPDR period, microangioma, hemorrhage, and exudation appear in the retina, while the PDR period is characterized by neovascularization, fibrosis, and proliferation. This syndrome is the ultimate destination of most cardiovascular diseases and the most important cause of death. It seriously threatens people's lives. With the aging of the population and the increase of the survival rate of myocardial infarction, it has become the cardiovascular disease with the fastest incidence rate. The method of constructing intelligent medical monitoring system is proposed to better study and observe the efficacy of trimetazidine combined with metoprolol in elderly patients with coronary heart disease complicated with heart failure and the effect of myocardial remodeling. Therefore, the intelligent nursing system is planned and developed as the main application of postoperative patients, intensive care patients, and chronic disease patients. It can realize the continuous measurement of vital signs parameters such as heart rate, blood oxygen, body temperature, and blood pressure, so as to carry out efficient monitoring and adjuvant treatment for patients. The whole process is small in size, complete in operation, and easy to move. With the advent of LoRa wireless technology, remote monitoring continued, and network services became more widespread [2]. The whole frame is shown in Figure 1.

## 2. Literature Review

Septianingrum and Susanto stated that currently, heart disease remains the leading cause of death and disability in industrialized countries [3]. Although treatment and surgery for heart disease have led to rapid growth and improved survival of heart disease patients, there are still a considerable number of patients with advanced ischemic cardiomyopathy who are not suitable for revascularization treatment. Sun et al. believe that drug therapy has become a supplementary treatment measure to replace interventional therapy for such patients [4]. Chen et al. said that the traditional treatment of ischemic cardiomyopathy heart failure is the same as that of heart failure caused by various reasons. It mainly changes hemodynamic parameters and reduces myocardial oxygen consumption, but the mortality of heart failure continues to increase. Optimizing myocardial energy metabolism can reduce the damage caused by myocardial ischemia and improve myocardial function without affecting hemodynamic parameters [5]. Pavlova believes that due to the interaction between cardiac metabolism and cardiac function, changing the conversion of cardiac metabolites from fatty acids to glucose is helpful to improve cardiac systolic function and delay the process of pump failure, which may become a new therapeutic target to improve the cardiac function of failing heart [6]. Mikhailova et al. said trimetazidine is one of the metabolic regulating drugs widely used in clinic. As a drug to improve energy metabolism of ischemic myocardium, it has been widely recognized by people in ischemic heart disease [7].

Reutersberg et al. say that Shengmai injection is based on the old Shengmai Powder formula. The main products are red ginseng, *Ophiopogon japonicus*, and *Schisandra chinensis* which are responsible for replenishing qi, nourishing yin, solidifying yin and removing it, replenishing water, and stopping the sweating. It is most commonly used to treat myocardial infarction, cardiogenic shock, and septic shock [8]. Wang et al. summarized the reports on the clinical application and research of Shengmai injection according to the relevant literature and summarized the following effects on hemodynamics. Shengmai injection has different effects on blood pressure in different states, reflecting the two-way regulation of blood pressure [9]. Zhang et al. stated that in animal experiments, Shengmai injection decreased the blood pressure of normal anesthetized dogs and increased the arterial pressure of rabbits with hemorrhagic shock during resuscitation [10]. While adjusting blood pressure, the heart rate does not increase, the cardiac output does not change or increase, the left ventricular filling pressure does not change or decrease, and the peripheral resistance decreases in varying degrees, suggesting that Shengmai injection increases the cardiac stroke volume, and the myocardial oxygen consumption does not increase or decreases slightly. Due to the unique pharmacological effect of Shengmai injection, it is different from some positive inotropic drugs and general vasodilators. As a “cardiotonic drug”, it can improve cardiac output and cardiac pumping function under different load conditions. As a “vasodilator”, it has no effect of reflex heart rate acceleration. In the experiment, it was found that when the Shengmai was injected into the right atrium too fast, the urine output decreased, the left ventricular filling pressure increased, and the heart beat slowed down. Scientists believe that high concentrations of Shengmai injection can inhibit heart function.

## 3. Method

### 3.1. Design of Front-End Monitoring System

*Part I: System Initialization*. The initialization module of LoRa, LoRa sensor, and LoRa base station.

*Part II: Algorithms for Signal Reception and Symbol Parameters*. The max31002 sensor detects the pulse wave of the fingertip, calculates the oxygen saturation of the blood by destroying the peak frequency and peak data of the pulse wave between the signal and the infrared light, and monitors the peak point of the pulse signal; the pulse wave conduction time is calculated by extracting the characteristic points of the pulse peak position irradiated by the same light source at the radial artery and fingertip, so as to calculate the blood pressure parameters [11]. MLX90614 infrared temperature sensor reads the RAM address and calculates the body temperature value by using the formula. The collected original pulse signal is preprocessed and the eigenvalue is extracted, which can realize the calculation of heart rate, blood oxygen, and blood pressure. The blood oxygen calculation model also needs to adjust its formula. Blood pressure is expressed according to the mathematical relationship between blood pressure and pulse wavelength (PTT), the continuous monitoring of blood pressure can be realized by determining parameters A and B through the proposed individualized parameter calibration method [12].

*Part III: OLED Display and LoRa Base Station*. The main controller sends physical information to the OLED during operation. At the same time, the time data is sent to the LoRa central station through the LoRa sending module, and then sent from the LoRra central station to the medical center (PC clinic), which can be provided for medical staff. Treat patients with kindness [13].

### 3.2. LoRa Base Station Program Design

LoRa is a kind of LPWAN, which can realize wireless network transmission with longer distance and lower power consumption and solve the problem that low power consumption and long distance cannot be used at the same time. LoRa needs to adjust the transmission speed (SF), encoding speed (CR), and signal bandwidth (BW) during the wireless connection. The distribution spectrum is determined by the number of characters sent to the 6-12 bit data. The larger the spread spectrum factor, the slower the transmission rate and the larger the network range [14]. The encoding rate is the distribution of values in the data stream. If the number of codes is K/N, the encoder generates *n* data for all *k* significant data, where *n* − *k* is redundant [15]. The larger the signal bandwidth, the faster the transmission rate, the shorter the transmission time, and the lower the reception sensitivity. The controller first initializes the UART port, then sets the spread spectrum factor, coding rate, and signal bandwidth transmitted by the LoRa wireless communication module, then receives data through the UART port, and finally transmits the data.

### 3.3. Programming of OLED Display Module

The system selects 0.96 inch OLED as the information display module. The module drives the chip SSD1306 and uses PC bus to transmit data through serial clock (SCL) and serial data line (SDA). PC protocol stipulates that there are three signal types during data transmission: start signal, stop signal, and reply signal [16]. The timing diagram of data transmission is shown in Figure 2.

The flow chart of OLED data display is shown in Figure 3.

### 3.4. Acquisition and Processing of Pulse Wave Signal

Pulse sensor is used on the blood pressure monitoring module to collect signals. Because the pulse wave signal belongs to physiological signal, its amplitude is small and easy to be disturbed by all kinds of noise. Therefore, low-pass filter and amplifier are added at the back end of the sensor, which can make the signal better collected by MCU ad.

At present, the most common applications of signal preprocessing include moving medium filtering, adaptive filtering, and wavelet transform filtering. [17]. Among them, wavelet transform denoising can well protect useful signal spikes and abrupt signals. Therefore, the software filtering of pulse wave signal is realized by the Mallat algorithm of wavelet transform. Because the pulse signal collected by the sensor is denoised to a certain extent, the waveform is smooth, and there is almost no high-frequency noise (including power frequency interference), the influence of baseline drift is mainly removed in the signal processing part. Wavelet Mallat algorithm is proposed by S. Mallat on the basis of summarizing a large number of previous work experiences. Combined with the tower algorithm, a fast algorithm for signal tower multiresolution analysis and reconstruction is proposed, which is called the Mallat algorithm, making wavelet multiresolution analysis practical [18].

In the Mallat algorithm, the selection of wavelet basis is very important. Because the signal characteristics presented by different wavelet basis functions are different, it is necessary to select the appropriate wavelet basis function. Usually, the selection is based on the wavelet base similar to the signal waveform to be processed. Another key factor in the Mallat algorithm is the selection of threshold. If the threshold is too small, the variance will be too large and the denoising is not complete; if the threshold is too large, it will lead to the loss of singularity of the signal and lead to deviation [19]. In the selection of threshold, the general threshold given by Donoho et al. is shown in Formula (1):

(1) $$\begin{array}{c} \lambda =\delta \sqrt{2\log\left(N\right)}. \end{array}$$

In practical application, with the increase of the number of decomposition layers, the amplitude of noise will gradually decrease. For the processing of physiological signals, the general threshold is improved with reference to the research results in this field. Therefore, the threshold of each layer can be expressed as shown in formula (2):

(2) $$\begin{array}{c} \lambda \left(j\right)=\frac{\delta \sqrt{2\log\left(N\right)}}{\log\left(j+1\right)}, \end{array}$$

where *j* represents the decomposition process. Once the starting point is determined, the starting point needs to be measured (how the starting point is applied to the wavelet coefficients). The two most used startups are the hard work and soft work segments. The basic math problem is in formula (3):

(3) $$\begin{array}{c} W_{h}\left(j,k\right)=\left\{\begin{array}{cc} W\left(j,k\right), & \left|W_{h}\left(j,k\right)\right|>\lambda ,\\ 0, & \left|W_{h}\left(j,k\right)\right|\leq \lambda , \end{array}\right. \end{array}$$

where *W*(*j*, *k*) is the wavelet coefficient after signal wavelet decomposition. The processing method of hard threshold function is to directly set the wavelet coefficients whose absolute amplitude is less than or equal to the set threshold to zero, while retaining the wavelet coefficients whose absolute amplitude is greater than the threshold. The mathematical expression of soft threshold function is shown in formula (4):

(4) $$\begin{array}{c} W_{s}\left(j,k\right)=\left\{\begin{array}{cc} \mathrm{sign}W\left(j,k\right)\left(\left|W_{h}\left(j,k\right)\right|-\lambda \right), & \left|W_{h}\left(j,k\right)\right|>\lambda ,\\ 0, & \left|W_{h}\left(j,k\right)\right|\leq \lambda . \end{array}\right. \end{array}$$

It can be seen from the display that the operation of the eye is not as simple and rude as the hard start on the small-amplitude wavelet coefficients, but to suppress all the wavelet coefficients. Through the adaptive calculation of formulas (1), 3, and 4, the threshold is 0.3. The effect of soft and hard threshold method on the straight line is shown in Figures 4–6.

### 3.5. Acquisition of Heart Rate, Blood Oxygen and Body Temperature Parameters

*(1) Acquisition of Heart Rate*. Heart rate is the amount of time a person's heart beats at rest, which is also the number of times the pulse beats. Heart rate is calculated as the average of patterns on adjacent peaks of infrared light over K cycles. The calculation formulas is shown in formulas (5) and (6)[20]:

(5) $$\begin{array}{c} \text{peak}\_\text{interval}\_\text{num}=\frac{\sum_{i}^{k-1}\left({\text{peak}}_{i+1}-{\text{peak}}_{i}\right)}{k-1}, \end{array}$$

(6) $$\begin{array}{c} \text{heart}\_\text{rate}=\frac{fs}{\text{heart}\_\text{interval}\_\text{num}}\times 6, \end{array}$$

where peak_*i*_ = (1, 2, ⋯k_*i*_) represents the abscissa of the peak point of K cycles, and peak_interval_num represents the average value of the coordinates between adjacent peaks in K cycles. The heart rate acquisition process is shown in Figure 7.

*(2) Acquisition of Blood Oxygen Saturation*. The maximum and minimum values of the collected pulse wave signal are used to represent the DC and AC components, as shown in formulas (7)–(9):

(7) $$\begin{array}{c} I_{\text{AC}}=I_{\max}-I_{\min}, \end{array}$$

(8) $$\begin{array}{c} I_{\text{DC}}=\frac{I_{\max}+I_{\min}}{2}, \end{array}$$

(9) $$\begin{array}{c} R=\frac{\left(I_{\text{red }\max}-I_{\text{red}\min}\right)/\left(\left(I_{\text{red}\max}+I_{\text{red}\min}\right)/2\right)}{\left(I_{\text{ir }\max}-I_{\text{rir }\min}\right)/\left(\left(I_{\text{ir}\max}+I_{\text{ir }\min}\right)/2\right)}=\frac{\left(I_{\text{ir }\max}+I_{\text{ir }\min}\right)\times \left(I_{\text{red}\max}-I_{\text{red}\min}\right)}{\left(I_{\text{red}\max}+I_{\text{red}\min}\right)\times \left(I_{\text{ir }\max}-I_{\text{rir }\min}\right)}, \end{array}$$

where *I*_redmax_ is the pulse wave peak value collected by red LED irradiation, *I*_irmax_ is the pulse wave peak value collected by infrared LED irradiation, and *I*_rirmin_ is the pulse wave valley value collected by infrared LED irradiation. According to the Lambert Beer's law, the calculation formula of bleeding oxygen can be calculated, as shown in formula (10):

(10) $$\begin{array}{c} {SpO}_{2}=\left(\frac{E_{2}^{\lambda_{2}}}{E_{1}^{\lambda_{1}}-E_{2}^{\lambda_{1}}}\times \frac{I_{\text{AC}}^{\lambda_{1}}/I_{\text{DC}}^{\lambda_{1}}}{I_{\text{AC}}^{\lambda_{2}}/I_{\text{DC}}^{\lambda_{2}}}-\frac{E_{2}^{\lambda_{1}}}{E_{1}^{\lambda_{2}}-E_{2}^{\lambda_{2}}}\right)\times 100\%. \end{array}$$

The constant term of the above formula can be expressed by *A* and *B* and the above formula can be obtained as shown in formula (11):

(11) $$\begin{array}{c} {SpO}_{2}=\left(A\times R-B\right)\times 100\%. \end{array}$$

It can be seen from the above formula that the estimation model includes two empirical constants *A* and *B*. due to different manufacturers and detection locations, the two undetermined parameters are also different, so it is necessary to calibrate the blood oxygen parameters through experiments. At this stage, considering the cost and performance of the experiment, Yuyue YX301 finger-clip pulse oximeter is selected as the calibration device, and the *R* value is calculated by this system. The experiments were performed on 10 volunteers who exchanged human blood oxygen by holding their breaths. The experimental data are shown in Table 1.

According to the above experimental data, taking *R* value as the abscissa and blood oxygen value as the ordinate, the calibration parameters can be obtained through data fitting. As shown in Figure 8.

### 3.6. Blood Pressure Acquisition

The system determined the use of two PPG markers to obtain the activity of the heartbeat to determine the continuous monitoring of blood pressure [21]. Pulse signals at the fingertips and radial vein (wrist) are done accordingly. Subsequently, the result of combining the points of n cycles can be expressed as *X* and *Y*, as shown in formulas (12) and (13):

(12) $$\begin{array}{c} X=\overset{n}{\underset{i=1}{\sum }}x_{i}, \end{array}$$

(13) $$\begin{array}{c} Y=\overset{n}{\underset{i=1}{\sum }}y_{i}. \end{array}$$

The *X* and *Y* parts represent the abscissa equation of the *n* feature point of the radial artery and the pulse wave signal of the fingertip, respectively. In this way, the difference of *n* similarity features can be expressed, as shown in formula (14):

(14) $$\begin{array}{c} T=\frac{X-Y}{n}. \end{array}$$

To reduce the error, the difference between the pulse on time (PTT) *n* and the sum of the sampling time (Ts) can be given. The sampling rate of the system is 100 Hz. As shown in formula (15).

(15) $$\begin{array}{c} \text{PTT}=\bar{T}\times \text{Ts}. \end{array}$$

The first step in researching blood pressure algorithms is based on the relationship between pulse wave transmission and blood pressure. As shown in formula (16):

(16) $$\begin{array}{c} \text{PTT}=a+b\times \text{PTT}. \end{array}$$

Based on this principle, the polynomial absorption method is used to establish the structural relationship between pulse wave conduction and pressure, in order to find a wide range of blood pressure estimation model through data fitting. The following are the test steps: measure the blood pressure value of the model with a standard sphygmomanometer, calculate the running time of the pulse with a system sphygmomanometer, and record the data. Systolic and diastolic blood pressure measurements were selected as standard numerical criteria. Sixteen volunteers (10 males and 6 females; aged 24-26 years, healthy and nonviolent) were selected to measure blood pressure using a machine-type electric sphygmomanometer and a temporal pulse wave measuring machine. The tested object needs to sit still for 2~3 minutes and starts when the heart rate is stable. During the measurement, each blood pressure data group was measured 3 times, and the average value was taken. If the difference is greater than one measurement (greater than 8 mmHg), the measurement should be repeated. The average time for each measurement should be at least 2 minutes.

The main factor of coronary heart disease causing myocardial hypoxia, ischemia, and myocardial infarction is heart failure. Epidemiological studies have pointed out that with the aging of the Chinese population, the incidence of coronary heart disease, hypertension, and other cardiovascular diseases is increasing year by year. The incidence of heart disease complicated by heart failure is also gradually increasing. Trimetazidine is a commonly used drug for the treatment of coronary heart disease and angina pectoris. It can selectively inhibit the oxidation process, increase the metabolic process, and regulate the energy metabolism of myocardial cells. Studies have shown that trimetazidine can reduce the release of oxygen free radicals and endothelial cells, reduce the decrease in myocardial function caused by injury or apoptosis, and achieve the purpose of improving myocardial function.

In order to solve the problems existing in the process of measuring blood pressure with equation parameter equation, improve the measurement accuracy and intensity of measurement parameters, and facilitate everyone to use. After experimental comparison, the linear equation between pulse conduction time and blood pressure is used as the estimation model, and the proposed new individualized parameter calibration method is used to improve the calibration of fixed parameters.

Smart clinical trials were designed and implemented. Its main function which is the front-end monitoring module combines LoRa wireless communication to monitor the patient's blood pressure, heart rate, blood oxygen, and body temperature in real time. Measurement systems and blood pressure monitors are responsible for collecting and transmitting data. Medical monitoring platforms identify the real-time presence of multiple malignancies and manage and maintain patient data [22]. It can be applied not only to hospital scenes but also to community medicine, family medicine, or personal health monitoring. The system realizes the characteristics of miniaturization of monitoring equipment, high measurement accuracy, convenient operation, and wireless data transmission and provides more convenient and efficient conditions for medical personnel. The software design of intelligent monitoring system is completed. Denoise the collected pulse wave raw data, remove the baseline influence through the wavelet Mallat algorithm, and then extract the pulse wave feature points by combining time-domain features and first-order differentiation [23]. The heart rate data is calculated by preprocessing the pulse signal and identifying the characteristic points; through the calibrated blood oxygen calculation model, the blood oxygen monitoring is realized; the radiation value of human body can be obtained through the detection of body temperature; the pulse wave conduction time is determined by collecting two pulse wave signals. According to the linear relationship with blood pressure, combined with the individualized parameter calibration method, the exclusive blood pressure calculation expression is finally determined to realize the continuous monitoring of blood pressure [24].

Oxidative stress injury is considered to be an important mechanism that leads to coronary heart disease and heart failure. Excessive reactive oxygen species act directly on unsaturated fatty acids in the body, leading to lipid peroxidation and resulting in oxidative stress injury and oxidative stress, and the body chronic inflammatory response is an important factor in the damage of vascular endothelial structure and function, and it is also the main reason for the increase in disease. The results of this study also showed that the patients in the observation group treated with trimetazidine combined with metoprolol had more significant improvement in LVEF, LVEDd, and LVESd.

## 4. Results and Conclusions

60 patients with ischemic cardiomyopathy and heart failure were hospitalized or outpatient in a hospital from February 2020 to October 2021. The inclusion criteria are (1) age > 50 years old. (2) According to the classification standard of cardiac function of the Heart Association, the cardiac function is grade, the left ventricular ejection fraction examined by echocardiography is, there is a clear history of myocardial infarction, or there are multiple lesions confirmed by coronary artery or coronary angiography. Inclusion criteria included acute pulmonary edema, severe hypertension, severe arrhythmia, severe liver and kidney failure, and acute cerebrovascular disease. They are divided into two groups: the management team and the medical team. There are 30 board members, 18 males and 12 females, aged 55-772, with an average age of 66.5 years and 30 outpatients included 16 males and 14 females, ages 56-774, with an average age of 67 years. Before treatment, there was no difference in age, sex, left ventricular injection portion, and cardiac function between the two groups [25].

B-type natriuretic peptide (BNP) is a polypeptide synthesized in cardiomyocytes. It is produced when ventricular volume increases, cardiac pressure load increases, and ventricular wall muscle tension increases. It has the functions of natriuresis, diuresis, and vasodilation and a natural antagonist of the renin-angiotensin-aldosterone system (RAAS system) and the sympathetic nervous system.

All patients received digitalis, angiotensin converting enzyme inhibitors, aldosterone antagonists, receptor blockers, and diuretics. The treatment group was given 20 mg 3 times/d as routine treatment. The duration of the exam is 2 months. All patients were screened every 2 months. Blood pressure and heart rate were measured on the first day and two months after the meal, and electrocardiogram, cardiac function, and color Doppler echocardiography were performed. Left ventricular and diastolic diameter, left ventricular fractional excretion, liver function, renal function, blood glucose, blood lipids, and hematuria were measured daily by biochemical parameters [26]. Left ventricular systolic function was measured with a color Doppler ultrasound. Blood pressure, heart rate, heart function, electrocardiogram, left ventricular and diastolic diameter, left ventricular secretion fraction, liver function, kidney function, blood sugar, blood lipid levels, and hematuria before and after treatment as usual. It should be noted that the improvement in cardiac function after treatment is greater than level 2, the improvement in cardiac function after treatment is very good, and the improvement of heart after treatment without improvement or serious. The evaluation standard of ECG curative effect is that the resting ECG ischemic change returns to normal, the ST segment of ECG ischemic decline rises by more than 0.1mv, or the inverted T wave of main lead becomes shallower by more than 50%, or the flat T wave becomes upright T wave, which is effective, and it is invalid if it fails to meet the above standards [27].

All measurements are presented as a ± variance model, and analysis of variance was used for subgroup and control comparisons. A *T* test was used for each measurement before and after treatment. All statistical data were analyzed using SPSS 160 software (*P* < 0.05).

### 4.1. Results

#### 4.1.1. Comparison of Changes in Cardiac Function in Both Groups Before and After Treatment

Left ventricular and diastolic LVEDD improved significantly compared with control group and postoperative group. The left ventricular ejection portion of the left ventricular septum was higher in the control and postoperative group than in the preoperative group. The improvement in the post-treatment group was significantly higher than that in the control group as shown in Table 2, Figures 9 and 10.

#### 4.1.2. Comparison of Clinical Efficacy

In the treatment group, 16 cases were positive, 10 were positive, and 4 were negative. The overall success rate was 86%. On the board, 13 passes are good, 9 are good, and 8 are bad. The overall success rate was 73%. The outcomes and overall outcomes of the two treatment groups were significantly better than those of the control group (*P* < 0.005) as shown in Table 3.

#### 4.1.3. Comparison of ECG Between the Two Groups After Treatment

In the treatment group, 15 cases were positive, 10 were positive, and 4 were negative. The overall success rate was 83%. On the board, 12 were excellent, 12 were positive, and 6 were negative. The overall success rate is 80%. The average outcome and summary of the two treatment groups were significantly better than those of the control group (*P* < 0.005), as shown in Table 4.

#### 4.1.4. Comparison of Blood Pressure and Heart Rate in the Pre- and Posttreatment groups

There was no difference in blood pressure and heart rate in the treatment group before and after treatment (*P* < 0.005). Trimetazidine does not affect hemodynamics as shown in Table 5.

No abnormality was found in blood glucose, blood lipid, liver function, renal function, and hematuria in the two groups after treatment.

Currently, heart disease is the leading cause of death and disability in industrialized countries. Although there is an increase in heart disease patients and their survival with treatment and surgery, many patients with ischemic cardiomyopathy are unable to perform revascularization [28]. Therefore, drug therapy has become a supplementary treatment measure to replace interventional therapy for these patients. The traditional treatment of ischemic cardiomyopathy heart failure is the same as that of heart failure caused by various reasons. Optimizing myocardial energy metabolism cannot affect hemodynamics, reduce the damage caused by myocardial ischemia, and improve myocardial function. The aim of this study was to evaluate the efficacy of triamcinolone acetonide in the treatment of ischemic cardiomyopathy and heart failure in the short term, which is better than therapeutic.

Inflammatory factors play an important role in the onset of heart failure, and the degree of inflammatory response stress is closely related to myocardial function and disease severity. The results of this study showed that the inflammatory factors in the observation group treated with trimetazidine combined with metoprolol The degree of decline in the level is more obvious, indicating that the combination of the two drugs can effectively inhibit the release of inflammatory factors, reduce the body's inflammatory response stress level, improve the cell environment, and reduce myocardial cell damage. The specific reasons still need to be further explored.

Chronic heart failure refers to the decline of myocardial contractility, so that the cardiac output cannot meet the needs of body metabolism, insufficient blood perfusion of organs and tissues, and the performance of monthly circulation and or systemic circulation blood addiction at the same time. The decisive mechanism of heart failure is ventricular remodeling. The decrease in the number of cardiomyocytes can reduce the contractility of myocardium, lead to the occurrence of myocardial infarction, and increase the load of viable cardiomyocytes, ventricular remodeling, and progressive deterioration. Studies have shown that there is an increase in apoptotic cardiomyocytes in the elderly, hypoxia, ischemia-reperfusion, myocardial infarction, and hypertrophic cardiorenal disease. The apoptosis of cardiac cells in patients with end-stage heart failure is times higher than that in normal people. In traditional Chinese medicine, heart failure is divided into five categories: “palpitations,” “asthma,” “edema,” “erectile,” and “phlegm-drinking”. These conditions recur and worsen over time. The main pathogenesis is deficiency, addiction, and drinking. Although it cannot communicate with the heart, moon, spleen, and kidney, its central qi deficiency is the most morbid variation. Since the heart does not contract, changes in RIC affect our lungs, spleen, and kidneys, and the liver is also affected.

### 4.2. Conclusion

The evaluation of myocardial changes and efficacy of trimetazidine combined with metoprolol in adults with congestive heart failure has been established. It can solve the problem of heart disease, meet the needs of shadow treatment of chronic diseases, make the difficulties of heart disease better, and improve the treatment effect of cardiovascular disease. Shengmai injection was replaced by a more form of Sanmai Changjing, an ancient Chinese herbal medicine. Maimendong plus Chuang Kong and ginseng are the two flavors of Shengmai injection. Shengmai injection is composed of red ginseng, *Ophiopogon japonicus*, and *Schisandra chinensis*. It can improve the energy generation and protein generation of heart failure myocardium, eliminate oxygen free radicals, inhibit lipid peroxidation, and enhance the low cellular immunity. It can improve the whole body and heart circulation, increase myocardial blood supply, reduce the load before and after the heart, protect the structure and function of damaged cardiomyocytes, prevent and delay the role of cardiomyocyte remodeling, so as to strengthen the myocardial contractility of patients with heart failure, improve the ability of myocardial hypoxia resistance, expand coronary artery and antiarrhythmia, and improve and protect cardiac function. At present, it has been widely used in the treatment of heart failure, tike, and other diseases.

The form of energy used by the heart is ATP, but ATP is rarely stored in the myocardium and must be synthesized in time. In a normal and healthy heart, 60%-90% of the energy required for myocardial activity comes from mitochondrial fatty acid metabolism, and the remaining 10%-40% comes from carbohydrates. After being absorbed by cells, fatty acids are transported into mitochondria through carnitine lipophthalein transferase I and enzyme II, that is, they are oxidized by *β* to produce acetylphthalein coenzyme A, and then recycled by tristate to produce ATP. The main sources of carbohydrates are glucose, lactic acid, and ketones. Myocardial glucose uptake generates pyruvate through glycolysis, and the absorbed lactic acid generates pyruvate through the action of lactate dehydrogenase. Pyruvate finally generates acetaldehyde coenzyme A under the action of pyruvate dehydrogenase, and then ATP is produced through trispinate cycle. Under the same oxygen supply conditions, fatty acids produce more energy than carbohydrates, but the oxygen utilization rate is low. To produce the same amount of ATP, fatty acids consume about 10% more oxygen than carbohydrates. This is particularly important when oxygen becomes a restrictive factor in oxidative metabolism. When the myocardial blood flow decreases by 20% -60%, the anaerobic glycolysis of glucose increases transiently, and the oxidation rate of free fatty acids decreases, but free fatty acids are still the main energy supply of myocardium. When the myocardial blood flow is reduced by more than 70% and the myocardial energy supply is still dominated by fatty acids, glycolysis will further increase, resulting in lactic acid accumulation and severe damage or complete loss of myocardial systolic function. When the blood flow is completely blocked, the intake of fatty acids stops completely, and glycolysis becomes the only energy source of cardiomyocytes. In the case of continuous hypoxia, the myocardium still takes fatty acids as the main source of energy, which will have an adverse effect. In the case of hypoxia, supplying energy in the way of high oxygen consumption will further aggravate the myocardial hypoxia. Fatty acids can inhibit the aerobic oxidation of glucose and reduce the production of ATP through PDH inhibition. A large amount of lactic acid accumulation, hydrogen ion accumulation, and pH value declination inhibits myocardial systolic function. The accumulation of intermediate metabolites of free fatty acids impairs the function of cell membrane. The etiology of ischemic myocardium the persistence of myocardial ischemia and hypoxia leads to the decrease of myocardial blood and oxygen supply, the increase of free fatty acid oxidation, the increase of energy consumption, the decrease of glucose metabolism, and the decrease of ATP production. Optimize myocardial energy metabolism, increase glucose metabolism, reduce free fatty acid oxidation, shift the oxidative metabolic substrate from free fatty acid to glucose, and use limited oxygen to produce more ATP. This study shows that trimetazidine combined with conventional heart failure drugs can increase muscle contractility and improve cardiac function in patients with ischemic cardiomyopathy without affecting hemodynamics. It was found that MCC950 can inhibit high glucose-induced damage of human retinal vascular endothelial cells, and the anti-inflammatory mechanism of MCC950 was verified to inhibit the activation of NLRP3 inflammasome by down-regulating NEK7-NLRP3 interaction.

## Figures and Tables

**Figure 1:** Overall framework of intelligent monitoring system.

**Figure 2:** PC data transmission sequence diagram.

**Figure 3:** Data display flow chart.

**Figure 4:** Original signal.

**Figure 5:** Effect of hard threshold.

**Figure 6:** Effect after applying soft threshold.

**Figure 7:** Heart rate acquisition flow chart.

**Figure 8:** Fitting diagram of blood oxygen calibration experiment.

**Figure 9:** Comparison before and after treatment (*P* < 0.0001).

**Figure 10:** Comparison before and after treatment (*P* < 0.001).

**Table 1:** Blood oxygen calibration experimental data.

Experiment number	1	2	3	4	5	6	7	8	9	10
The system measures the *R* value	0.6425	0.5818	0.5902	0.6284	0.7218	0.7024	0.6614	0.6841	0.5772	0.5546
YX301 measured blood oxygen	96%	98%	98%	97%	94%	94%	96%	95%	99%	99%

**Table 2:** Changes of various indexes of cardiac function in the two groups before and after treatment.

Group	Number of cases	Left ventricular end diastolic diameter (mm)		Ejection fraction (%)	
		Before treatment	After treatment	Before treatment	After treatment
Treatment group	30	56.97 ± 2.761	52.73 ± 3.618^∗∗^^#^	35.26 ± 5.328	39.20 ± 6.346^∗^^#^
Control group	30	55.91 ± 2.438	53.55 ± 2.315^∗^	36.42 ± 4.756	37.51 ± 6.374^∗^

**Table 3:** Comparison of the therapeutic effects of the two groups before and after heart failure treatment.

Group	Efficacy of heart failure			
	Remarkable effect	Effective	Invalid	Total effective rate
Treatment group	16 (53)	10(33)	4 (14)	26 (86)
Control group	13 (43)	9 (30)	8 (27)	22 (73)

**Table 4:** Comparison of ECG between the two groups before and after treatment.

Group	ECG changes			
	Remarkable effect	Effective	Invalid	25 (83)
Treatment group	15(50)	10(33)	5 (17)	26 (86)
Control group	12(40)	12(40)	6 (20)	22 (80)

**Table 5:** Comparison of blood pressure and heart rate in the treatment group before and after treatment.

Number of cases	Mean systolic blood pressure (mmHg)		Average heart rate (beats/min)	
	Before treatment	After treatment	Before treatment	After treatment
30	135 ± 15	128 ± 18	80 ± 6	81 ± 4

## Data Availability

No data were used to support this study.
